This article has been retracted.

# MicroRNA-20b (miR-20b) Promotes the Proliferation, Migration, Invasion, and Tumorigenicity in Esophageal Cancer Cells via the Regulation of Phosphatase and Tensin Homologue Expression

**DOI:** 10.1371/journal.pone.0164105

**Published:** 2016-10-04

**Authors:** Bin Wang, Jie Yang, Bin Xiao

**Affiliations:** 1 Department of Gastroenterology, Renmin Hospital, Hubei University of Medicine, Shiyan, 442000, Hubei Province, China; 2 Department of Medical Care Center, Renmin Hospital, Hubei University of Medicine, Shiyan, 442000, Hubei Province, China; 3 Ultrasonic Imaging Division, Renmin Hospital, Hubei University of Medicine, Shiyan, 442000, Hubei Province, China; Michigan State University, UNITED STATES

## Abstract

Increasing evidence has indicated that many microRNAs participate in the development and progression of esophageal cancer and gene expression regulation. MicroRNA-20b (miR-20b) has been reported to be aberrantly expressed in various cancers, but its exact role in esophageal cancer cells remains unclear so far. Therefore, we detected the levels of miR-20b in esophageal tumor tissues and their adjacent normal tissues, and various esophageal cancer cell lines by qRT-PCR. We also explored the effects of miR-20b on cell proliferation, migration, invasion and tumorigenicity of esophageal carcinoma cells through transfection with miR-20b mimics or inhibitor to upregulate or downregulate miR-20b expression in the esophageal cancer cells Eca-109 and KYSE-150, respectively. Additionally, the 3'-untranslated region (3'-UTR) of phosphatase and tensin homologue (PTEN) binding with miR-20b was analyzed by dual-luciferase reporter assays. The results indicated that miR-20b expression level in esophageal tumor tissues was significantly increased compared with their neighboring normal tissues, but its expression was inverse with PTEN protein expression. Luciferase assays confirmed that the 3'-UTR of PTEN was a target of miR-20b in esophageal cancer cells. MiR-20b upregulation promoted cell proliferation, migration, invasiveness, and tumor growth, and decreased apoptosis, and reduced PTEN protein level but not mRNA expression in Eca-109 cells. Conversely, downregulation of miR-20b suppressed these processes in KYSE-150 cells, and enhanced PTEN protein expression. These data indicate that miR-20b plays important roles in tumorigenesis of esophageal cancer possibly via regulation of PTEN expression, and it may be a potential therapeutic target for esophageal cancer treatment.

## Introduction

Esophageal carcinoma is one of the most malignant tumor types and represents the sixth leading cause of cancer death [1], and it is generally diagnosed at a late stage, and is associated with a poor prognosis with a five-year survival of less than 10% [2]. Increasing studies indicate that a poor survival rate in esophageal cancer patients is highly associated with a frequent local invasion and distant metastasis [3,4]. However, many molecular events involved in cell malignant proliferation, migration, invasion, and metastasis in the esophageal carcinoma cells have been identified, exact molecular mechanisms underlying these processes remain incomplete.

MicroRNAs (miRNAs, miRs) are small noncoding RNA molecules that regulate gene expression by mRNA degradation or translational repression through imperfect paring at the 3'-end of untranslated regions (UTRs) [5]. Increasing studies indicate that microRNAs participate in various biological processes, such as cell proliferation, differentiation, apoptosis, metabolism, and tumor genesis [6,7]. Recent data indicate that aberrant miRNA expression is often involved in cancer development from initiation to metastasis in various cancers including esophageal carcinoma [8]. Current evidence supports that miRNAs can served as either tumor suppressors or oncogenes [9,10].

Over the past few years, many deregulated miRNAs including miR-20b were found by using microarray analyses in various cancers [11,12]. Previous studies have demonstrated that miR-20b expression level is higher in the brain metastases of breast cancer patients, compared to primary breast tumors as well as the patients without brain metastasis, and miR-20b can induce colony formation and invasiveness of breast cancer cells [13]. Additionally, other studies indicated that miR-20b expression was upregulated in gastric cancer tissue compared with normal mucosa, and was positively correlated with advanced lymph node metastasis [14]. MiR-20b was also reported to favor the survival of tumor cell through the regulation of hypoxia-inducible factor-1 alpha (HIF-1 alpha) and vascular endothelial growth factor (VEGF) expression [15]. These studies suggested that miR-20b possibly plays an important role in the maintenance of tumor cell survival, invasion and metastasis. However, its expression and functional role in the esophageal cancer cells remain unclear. Therefore, in this study, we detected the levels of miR-20b expression in the esophageal tumor tissues and their neighboring normal tissues, and investigated the functional role of miR-20b on esophageal cancer cells. Our findings indicated that miR-20 expression promoted cell proliferation, migration, invasiveness and tumor growth in esophageal cancer cells. Additionally, we confirmed that miR-20b directly targeted the 3'-UTR of PTEN, and regulated PTEN protein expression. These results demonstrate that miR-20b is a potential therapeutic target for the treatment of esophageal cancer.

## Materials and Methods

### Tissue samples and ethics statement

A total of 38 cases of esophageal tumor tissues were obtained from patients collected at Renmin Hospital, Hubei University of Medicine. The matched normal tissues were obtained from adjacent tissues that were located more than 3 cm away from the tumors. The tumors were further confirmed by pathologists, and classified according to World Health Organization classification. All patients have not received any therapy before our research. This study was reviewed and approved by the Human Research and Ethical Committee of Renmin Hospital, Hubei Medical University. The written informed consent was obtained from every participant who involved in this study. The clinicopathological characteristics and parameters are shown in Table 1.

**Table 1:** Association between miR-20b expression and clinicopathological features of esophageal cancer patients.

Variables	Patients (n = 38)	Expression of miR-20b (Mean ± SEM)	*P*-value
**Age (years)**			
**≤ 60**	16	2.098 ± 0.524	0.875
**> 60**	22	2.212 ± 0.489	
**Gender:**			
**Male**	26	2.310 ± 0.573	0.391
**Female**	12	2.102 ± 0.804	
**Tumor size (cm):**			
**≤ 4**	23	2.115 ± 0.710	
**> 4**	15	2.387 ± 0.663	0.352
**Degree of differentiation:**			
**Highly and moderately**	20	1.799 ± 0.705	0.030*
**lowly**	18	2.354 ± 0.594	
**Invasion depth:**			
**T1 + T2**	22	2.051 ± 0.594	0.041*
**T3 + T3**	16	2.495 ± 0.513	
**TNM stage:**			
**Stage I + II**	25	1.883 ± 0.648	
**Stage III + IV**	13	2.426 ± 0.712	0.025*
**Metastasis**			
**Positive**	12	1.804 ± 0.659	0.037*
**Negative**	26	2.349 ± 0.583	

*P < 0.05 was considered to be a statistically significant difference.

TNM, tumor node metastasis.

### Cell culture and reagents

Human normal esophageal cell line Het-1A, and human esophageal carcinoma cell lines TE-1, Eca-109, EC9706, KYSE-150, and SKGT-5 were obtained from Cell Bank of Chinese Academy of Science (Shanghai, China), and were maintained in RPMI-1640 medium supplemented with 10% fetal bovine serum (Gibco, USA),100 IU/ml penicillin, and 100 μg/ml streptomycin, at 37°C in a humidified incubator with 5% CO_2_. MiR-20b mimics, miR-20b mimics negative control (miR-20b mimics-NC), miR-20b inhibitor, and miR-20b inhibitor negative control (miR-20b inhibitor-NC) were all purchased from Ribobio Company (Guangzhou, China). Annexin V-FITC/propidium iodide apoptosis detection kit was obtained from Promega Corporation (Madison, WI, USA). The primary antibodies against PTEN, p-Akt, Akt and β-actin were purchased from Cell Signal Technology (Beverly, MA, USA).

### Quantitative real-time RT-PCR (qRT-PCR)

Total RNA from cell lines Het-1A, TE-1, Eca-109, EC9706, KYSE-150, and SKGT-5 or tissue samples was separately extracted using a miRNA isolation kit (Takara, Japan), and followed by reverse transcription using one step PrimeScript^®^ miRNA cDNA synthesis kit (Takara) following the manufacturer’s instructions. The sequence-specific primers for mature miR-20b were as follows: forward, 5'-TGTCGACAAGCTTACACGA-3', reverse, 5'-GCTAGTCATGGTGCAAGA-3'. U6 small nuclear RNA was used to be a internal control and its sequence-specific primers were: forward, 5'-GCTCTCGCATCGCAGCA-3', reverse, 5'-CTCGGCTAGCGCTACTC-3'. The amplification of PCR was performed using the SYBR Premix Ex Taq (Takara) as described previously [16], on a LightCycler^®^ (Roche Diagnostics, USA). The amplification condition of PCR was as follows: 30 s at 94°C, and 40 cycles at 95°C for 5 s and 60°C for 20 s. Relative expression levels of were calculated by using the comparative 2^-ΔCT^ method [17].

### Cell transfection assay

Cell transfection was performed using Lipofectamine 2000 (Invitrogen Life Technologies, USA) according to the manufacturer’s instructions. For miR-20b functional analysis, its gain-of-function study was performed using miR-20b mimics (100 nM) and its negative control (miR-20b mimics-NC) (100 nM) on the Eca-109 cells. PTEN expressing vector was constructed by inserting PTEN cDNA into pcDNA3.1 vector, and was transfected into Eca-109 cells. Mock vector was used as the control for PTEN expression vector. On the other hand, the loss-of-function study was carried out with miR-20b inhibitor (100 nM) and its negative control (miR-20b inhibitor-NC) (100 nM) on the KYSE-150 cells. PTEN siRNA and its corresponding control siRNA were obtained from Invitrogen company (Carlsbad, CA USA), and also transiently transfected into KYSE-150 cells. There was a blank control without any transfection for each cell line. After transfection of 48 h, miR-20b expression level in the transfected cells was detected by qRT-PCR.

### Luciferase reporter assays

The region of human PTEN-3-'UTR targeted by miR-20b was predicted by miRanda (http://www.Microrna.org/) and TargetScan (http://www.targetscan.org/), and the direct targeted region was determined by cloning of the 3'-UTR seed regions and mutated seed regions into the pmiR-RB-REPORT luciferase reporter vectors (RiboBio Company, Guangzhou, China). The primers selected were as follows [18]: PTEN-wt-F:5'-CTAGAAATTAGGATTAATAAAGATGGCACTTTCCCGTTTTATTCCAGTT-3'; PTEN-wt-R: 5'-TTTAATCCTAATTATTTCTACCGTGAAAGGGCAAAATAAGGTCAAGATC-3'; PTEN-mut-F: 5'-CTAGAAATTAGGATTATTAAAGATGTTTGCACCCCGTTTTATTCCAGTT-3'; PTEN-mut-R: 5'-TTTAATCCTAATTATTTCTACAAACGTGGGGCAAAATAAGGTCAAGATC-3'. These constructs were named pmiR-PTEN-wt and pmiR-PTEN-mut, and transfected into esophageal carcinoma Eca-109 and KYSE-150 cells with miR-20b mimics, miR-20b inhibitors or negative control using Lipofectamine 2000. Luciferase activities were measured using the dual-luciferase reporter assay system (Promega, USA) 48 h after transfection according to the manufacturer’s instructions.

### Determination of mRNA expression levels of miR-20b and PTEN

Total RNA was isolated from the transfected Eca-109 and KYSE-150 cells 48 h after transfection. The expression level of miR-20b after transfection was determined using qRT-PCR as previously described. For the detection of PTEN mRNA expression level, qRT-PCR was also used in this study. Briefly, total RNA was reverse transcribed to cDNA using the SuperScript ^®^ RT kit (Invitrogen, USA), and PCR was performed on a LightCycler^®^. The specific primers for PTEN and glyceraldehyde-3-phosphate dehydrogenase (GAPDH) were as follows [18]: PTEN forward 5'-TTTGAAGACCATAACCCACCAC-3', and reverse 5'-ATTACACCAGTTCGTCCCTTTC-3'; GAPDH forward 5'-GGAGCCAAAAGGGTCATC-3', and reverse 5'-CCAGTGAGTTTCCCGTTC-3'. The programs of PCR amplification were as follows: 95°C for 5 min; 35 cycles of 94°C for 30 s, 55°C for 30 s, and 72°C for 30 s; and 72°C for 5 min. The mRNA level of PTEN was analyzed using the 2^-ΔCT^ method and normalized to GAPDH mRNA level.

### Western blotting

Total protein from esophageal cancer tissues, adjacent normal tissues, and cultured cells by RIPA buffer (ThermoFisher, USA) including protease inhibitors. After determination of protein concentration, equal amounts of total protein were separated by SDS-PAGE with 10% gel, and then transferred to polyvinylidene difluoride membranes (Millipore, USA). After blocking in 5% skimmed milk powder overnight at 4°C, the membranes were immunoblotted overnight at 4°C with primary antibodies against human PTEN, p-Akt, Akt (Cell Signaling Technology, USA), and β-actin served as the loading control, and followed by incubation with horseradish peroxidase-conjugated secondary antibodies for 1 h at room temperature. The signals were detected using an enhanced chemiluminescence reagent and system (Amersham Biosciences Corp., NJ, USA). The optical density of each band was quantified by using Quantity One software (Bio-Rad, Hercules, CA, USA).

### Cell viability assay

Cell viability was analyzed with 3-[4, 5-dimethylthiazol-2-yl]-2, 5-diphenyltetrazolium bromide assay (MTT assay). Briefly, the cells were plated in 96-well plates at a density of 1×10^4^ cells/well, and incubated for 24, 48, 72, and 76 h after transfection. 20 μl MTT (5 mg/ml solution in 1 × phosphate-buffered saline) was added to each well for incubation of 4 h at 37°C. After removal of supernatant, 150 μl of dimethyl sulfoxide (DMSO) was added to each well to dissolve the formazan. Absorbance value of each well was measured by an automated spectrophotometric plate reader (PerkinElmer, USA) at 570 nm. The experiments were independently performed in triplicate.

### Determination of apoptosis

Cellular apoptosis was determined with Annexin V-FITC and propidium iodide (PI) apoptosis detection kit. Briefly, Eca-109 and KYSE-150 cells were harvested 72 h after transfection, and washing twice with phosphate-buffered saline (PBS), and re-suspended in 500 μl of binding buffer containing 5 μl of Annexin V-FITC and 10 μl of PI for 30 min at room temperature in the dark, and measured with flow cytometry (BD Biosciences, USA). Cells were discriminated into viable (Annexin V-FITC and PI doubly negative), apoptotic (Annexin V-FITC positive and PI negative), and necrotic cells (Annexin V-FITC and PI doubly positive). Finally, the percentage of cellular apoptosis was analyzed with the CellQuest software.

### Wound healing assay

Migration abilities of Eca-109 and KYSE-150 cells after transfection were evaluated by wound healing assay as previously described [19], with some modifications. In brief, the cells were seeded in 6-well plates and grown to about 85% confluence, and a wound of each group was then created with a pipette tip, and washed with PBS to remove cell debris. After 24 h culture, the wounds were then observed and captured under an inverted microscope with 100 × magnification. Three randomly selected areas of each group were analyzed using Image J software to calculate the number of cells migrated into the wound areas.

### In vitro cell invasion assay

Cell invasion in vitro was evaluated by using Boyden transwell system with 12-well plates (BD Biosciences). Briefly, transwell membranes with 8 μm pore size were precoated with Matrigel (BD Biosciences) and allowed for solidification at 37°C. Eca-109 and KYSE-150 cells were respectively harvested at 48 h post- transfection, and resuspended into serum-free medium, and seeded into the upper chamber of transwell at 1 × 10^5^ cells per well in 200 μl of serum-free medium, and 0.6 ml of growth medium containing 10% fetal bovine serum was added into the bottom wells as chemoattractant. After 24 h incubation, the cells invaded through the membranes to the bottom wells were fixed in 75% ethanol, and then stained with hematoxylin and eosin solution, and counted from five randomly selected visual fields under an inverted microscope at 100 × magnification. The experiments were performed at least three times.

### In vivo tumorigenicity assays

Healthy athymic female BALB/c nude mice were purchased from the Shanghai Experimental Animal Center, and maintained at the Animal Center of Hubei University of Medicine. Sterilized food and water were available for the mice during the experimental period. The studies in mice were approved by the Animal Care and Use Committee (ACUC) of Hubei University of Medicine. The guidelines of ACUC were strictly followed in the whole process of animal studies. Eca-109 cells transfected with agomir-20b and its negative control (agomir-NC) or KYSE-150 cells transfected with antagomir-20b and its negative control (antagomir-NC) (5 × 10^6^ cells in 0.2 ml PBS) were respectively injected subcutaneously into the right flank of each mouse (5 mice/each group). Tumor size was determined one time with a caliper every 5 days until sacrifice. Tumor volume was calculated according to a formula *V* = π/6 (L × W)^3/2^ as described previously [20]. The *L* and W represented the length and width of tumors, respectively. After 40 days, the mice were sacrificed and the tumor tissues were weighed, and processed for qRT-PCR analysis and immunohistochemistry assays for miR-20b and PTEN expression level, respectively.

### Statistical analysis

All data were presented as the mean ± SD, and statistical analysis was performed with a software SPSS (version 13.0, Chicago, USA). The mean values of two groups or multiple groups were compared by Student’s *t* test or ANOVA. Differences with a value of *P* < 0.05 was considered statistically significant.

## Results

### Inverse level of miR-20b an PTEN protein in esophageal cancer and cells

The results of qRT-PCR analyses showed that expression levels of miR-20b were significantly up-regulated in esophageal cancer tissues compared to those in the corresponding adjacent normal tissues (Fig 1A). Based on the clinical information of patients, we found that the aberrant expression of miR-20b was related with the pathological stages including tumor differentiation degree, invasion depth, TNM stage, and lymph node metastasis in esophageal carcinoma patients (*P* < 0.05), although its expression had not significant correlation with age, gender and tumor size (*P* > 0.05) (Table 1). We further detected the expression levels of miR-20b in human normal esophageal cell line Het-1A, and human esophageal carcinoma cell lines (TE-1, Eca-109, EC9706, kyse-150, and SKGT-5). The results demonstrated that miR-20b expression was relatively higher in low differentiation cell lines (KYSE-150 and SKGT-5) than in high differentiation cell lines (TE-1, Eca-109, and EC9706) (Fig 1B). There was the lowest level of miR-20b expression in the normal esophageal cells Het-1 A and esophageal carcinoma cells Eca-109.

**Fig 1:** MiR-20b expression is associated with PTEN level. (A) The expression levels of miR-20b in 38 paired esophageal tumor tissues and their corresponding adjacent normal tissues were determined by qRT-PCR analyses. * *P* < 0.05. (B) qRT-PCR analyses of miR-20b expression in human normal esophageal cell line Het-1A, and human esophageal carcinoma cells including TE-1, Eca-109, EC9706, KYSE-150, and SKGT-5. The miR-20b expression was normalized by U6 expression that served as the internal control. * *P* < 0.05, and ** *P* < 0.01 compared with Het-1A. (C) The levels of PTEN protein between the esophageal tumor tissues (T) and corresponding adjacent normal tissues (N) were detected by Western blotting. (D) Quantitative analysis of PTEN protein expression that was normalized to β-actin. ** *P* < 0.01 compared with neighboring normal tissues. (E) The levels of PTEN protein in various cells were detected by Western blot analysis. (F) The relative levels of PTEN protein in various cells were normalized to β-actin. The data represent the mean ± SD (n = 3), * *P* < 0.05 compared with Het-1A.

Previous studies have exhibited PTEN is one of the target genes of miR-20b in breast cancer [5, 21]. Therefore, to investigate whether there is an association between PTEN and miR-20b expression, we randomly selected 5 paired clinical tumor tissues and adjacent normal tissues from 38 patients with esophageal cancer to detect the PTEN protein expression by Western blotting. The results demonstrated that the level of PTEN protein was reduced in human esophageal tumor tissues compared with neighboring normal tissues (Fig 1C and 1D). Additionally, a decreased level of PTEN protein in various esophageal cancer cells was observed compared with normal esophageal cells Het-1A (Fig 1E and 1F). These data suggest that the expression level of PTEN protein is negatively correlated with miR-20b expression in esophageal cancer cells and esophageal tumor tissues.

### MiR-20b binds to the 3'-UTR of PTEN

Based on above results of miR-20b expression in various cell lines, Eca-109 and KYSE-150 cells were chosen for the following functional studies of miR-20b through gain-of-function and loss-of function investigation, respectively. To investigate the potential sites targeted by miR-20b, available miRanda and TargetScan were used to predict the region of target gene. As shown in Fig 2A, PTEN is a putative target gene of miR-20b. Luciferase reporter assays were used to confirm that miR-20b directly targets PTEN. Further studies demonstrated that co-transfection of miR-20b mimics and pmiR-PTEN-wt markedly reduced the luciferase activities in Eca-109 cells and KYSE-150 cells but not that of the mutant reporter (Fig 2B and 2C), suggesting that miR-20b can directly bind to the 3'-UTR of PTEN.

**Fig 2:** MiR-20b directly targets the 3'-UTR of PTEN. (A) The position of miR-20b target site in 3'-UTR of PTEN mRNA predicted by miRanda and TargetScan. (B-C) Luciferase assays in Eca-109 cells (B) and KYSE-150 cells (C), and these cells were cotransfected with wt/mut-3'-UTR with miR-20b mimics or negative control (miR-NC). Luciferase activity was detected using dual- luciferase reporter assay system following the manufacturer’s instruction 48 h after transfection. The results were expressed as fold change relative to the negative control. The data represent the mean ± SD (n = 5). * *P* < 0.05, compared with the corresponding negative control.

### MiR-20b regulates PTEN expression at posttranscriptional level

To investigate the effect of miR-20b on PTEN expression level, Eca-109 and KYSE-150 cells were respectively transfected with miR-20b mimics or miR-20b inhibitor. The results indicated that transfection with 100 nM of miR-20b mimics in Eca-109 cells resulted in a significant increase in miR-20b expression as determined by qRT-PCR when compared to blank control or miR-20b mimics-NC (Fig 3A). On the contrary, KYSE-150 cells transfected with 100 nM of miR-20b inhibitor dramatically reduced miR-20b expression level as compared with the blank control or negative control (miR-20b inhibitor-NC) (Fig 3B). Further investigation showed that PTEN mRNA level was not significantly changed in both cell lines after transfection with miR-20b mimics or miR-20b inhibitor (*P* > 0.05) (Fig 3C and 3D). However, a downregulated level of PTEN protein was observed in the Eca-109 cells after transfection with miR-20b mimics (Fig 3E and 3F). In contrast, a marked increase of PTEN protein expression was found in the KYSE-150 cells after transfection with miR-20 inhibitor (*P* < 0.05). On the other hand, previous studies demonstrated that miR-20b plays an important role in PTEN/Akt signaling pathway carcinogenesis and the progression of esophageal cancer [22]. Accordingly, we determined the protein levels of Akt and its phosphorylated forms (p-Akt). The results showed that miR-20b mimics and miR-20b inhibitor did not alter the protein level of Akt in the Eca-109 and KYSE-150 cells, but miR-20b mimics significantly up-regulated the level of p-Akt compared with miR-20b mimics-NC in the Eca-109 cells. On the contrary, miR-20b inhibitor markedly reduced the level of p-Akt in the KYSE-150 cells.

**Fig 3:** MiR-20b inhibits PTEN protein expression and increases p-Akt level. (A-B) MiR-20b expression was detected by qRT-PCR. A sharp increase of miR-20b expression was observed in the Eca-109 cells transfected with miR-20b mimics (A), while KYSE-150 cells transfected with miR-20b inhibitor resulted in a significant decrease of miR-20b expression (B). (C-D) PTEN mRNA expression was determined by qRT-PCR, and the results indicated that these transfected Eca-109 cells (C) and KYSE-150 cells (D) had no alternation in PTEN mRNA level. (E) The representative images of Western blotting for PTEN, p-Akt and Akt protein expression. (F) Quantitative analysis protein levels of PTEN, p-Akt and Akt by normalization to β-actin. The data represent the mean ± SD (n = 3). * *P* < 0.05, compared with the corresponding blank control or negative control.

### MiR-20b promotes esophageal carcinoma cell proliferation

To further study the functional role of miR-20b on the growth of esophageal carcinoma cells, MTT assays was used to evaluate cell proliferation in the Eca-109 cells and KYSE-150 cells transfected with miR-20b mimics and miR-20b inhibitor, respectively. The results demonstrated that miR-20b overexpression significantly increased the proliferation of Eca-109 cells, whereas miR-20b inhibition suppressed the proliferation of KYSE-150 cells at 48, 72, and 96 h after transfection in comparison with the corresponding blank control or negative control (Fig 4).

**Fig 4:** Effects of miR-20b on the proliferation of esophageal carcinoma cells Eca-109 and KYSE-150 cells were transfected with miR-20b mimics and miR-20b inhibitor, respectively. Cell proliferation was evaluated by MTT assays after the indicated periods. (A) Transfection with miR-20b mimics promoted Eca-109 cell proliferation. (B) Transfection with miR-20b inhibitor suppressed KYSE-150 cell proliferation. The data represent the mean ± SD (n = 3). * *P* < 0.05, compared with blank control or negative control.

### MiR-20b attenuates apoptosis in esophageal carcinoma cells

Cell apoptosis was detected by flow cytometry 72 h after Eca-109 cells and KYSE-150 cells were transfected with miR-20b mimics and miR-20 inhibitor, respectively. As shown in Fig 5, the results showed that the percentage of apoptotic cells (Annexin V-FITC^+^/PI ^-^) was significantly reduced in miR-20b transfected Eca-109 cells compared to the blank control or negative control (*P* < 0.05). However, the forced overexpression of PTEN in the Eca-109 cells by transfection of its expressing vector increased cellular apoptosis. On the other hand, miR-20b expression downregulation by miR-20b inhibitor markedly increased apoptotic percentage in the KYSE-150 cells (*P* < 0.05). Silenced PTEN expression in the KYSE-150 cells using PTEN siRNA resulted in a decreased cellular apoptosis. These data suggest an anti-apoptotic function of miR-20b in esophageal carcinoma cells possibly through regulation of PTEN expression.

**Fig 5:** Effects of miR-20b on cellular apoptosis. Apoptotic percentage in Eca-109 cells or KYSE-150 cells was determined by flow cytometry through the double staining with Annexin V-FITC/ propidium iodide (PI). (A) Representative plots of flow cytometry detection for apoptosis. The percentage of apoptosis was shown in the bottom right quadrant. (B) Apoptotic percentage was quantified and expressed as fold change relative to the corresponding blank control. The data represent the mean ± SD (n = 3). *P < 0.05, ^#^*P* < 0.05, and ^△^*P* < 0.05.

### MiR-20b promotes the migration and invasion of esophageal carcinoma cells

To investigate the effects of miR-20b on the abilities of cell migration and invasion in the Eca-109 cells and KYSE-150 cells after transfection of 48 h, wound healing assay and in vitro Matrigel invasion assay were performed. The results demonstrated that overexpression of miR-20b significantly increased the abilities of cell migration and invasion in Eca-109 cells, whereas miR-20b expression downregulation suppressed KYSE-150 cell migration and invasiveness (Figs 6 and 7). On the other hand, the forced overexpression of PTEN in the Eca-109 cells reduced the abilities of cell migration and invasion. However, silenced PTEN expression in the KYSE-150 cells increased their abilities of cell migration and invasion. These findings suggest that miR-20b has a positive role in promoting esophageal carcinoma cell migration and invasiveness.

**Fig 6:** Wound healing assay. The ability of cell migration was evaluated by wound healing assay after transfection of 48 h. (A) Representative photographs taken at 0 and 24 h after a wound of each group was created by a pipette tip. (B) The number of cells migrated into wound areas was calculated and expressed as fold change relative to the corresponding blank control. The data represent the mean ± SD (n = 3). *P < 0.05, ^#^*P* < 0.05, and ^△^*P* < 0.05.

**Fig 7:** Transwell invasion assay. The ability of cell invasion in vitro was evaluated by Boyden transwell system with porous membranes that were pre-coated with Matrigel after transfection of 48 h. (A) Representative photographs taken at 24 h after the cells were seeded into the upper chamber of transwell, and the cells penetrated through the Matrigel and membranes were fixed in 75% ethanol and stained with hematoxylin and eosin solution. (B) The numbers of cells that penetrated through the membranes to the bottom wells was calculated at five randomly selected visual fields, and expressed as fold change relative to the corresponding blank control. The data represent the mean ± SD (n = 5). * *P* < 0.05, ^#^*P* < 0.05, and ^△^*P* < 0.05.

### MiR-20b expression promotes tumor growth in vivo

To investigate the effect of miR-20b on tumorigenicity of esophageal carcinoma cells in vivo, Eca-109 cells transfected with agomir-20b or negative control (agomir-NC), and KYSE-150 cells transfected with antagomir-20b and its negative control (antagomir-NC) were subcutaneously inoculated into nude mice, respectively.

The results demonstrated that Eca-109 cells transfected with agomir-20b promoted tumor formation and growth, produced a significant increase in the tumor size and average weight compared with agomir-NC group (Fig 8A). On the contrary, KYSE-150 cells transfected with antogomir-20b markedly suppressed tumor growth, and significantly reduced tumor volume and their average weight compared with the antagomir-NC group (Fig 8B and 8C). The results of qRT-PCR showed that miR-20b expression level was significantly up-regulated in the tumor tissues of agomir-20b group (Fig 8D). Inversely, a reduced level of PTEN protein expression in these tumor tissues was observed by immunohistochemistry (Fig 8E). On the other hand, the level of miR-20b expression was significantly down-regulated in the tumor tissues of antogomir-20b compared with its negative control. By contrast, the level of PTEN protein was up-regulated in these tumor tissues. These results indicated that miR-20b expression promoted esophageal tumor growth in vivo possibly regulation of PTEN protein expression.

**Fig 8:** MiR-20 expression promotes tumorigenicity of esophageal carcinoma cells in vivo. (A-B) Effects of agomir-20b (A) and antagomir-20b (B) on tumor volume in the xenograft model of nude mice. Female BALB/c nude mice were respectively inoculated with Eca-109 cells transfected with agomir-20b or its negative control (agomir-NC), and KYSE-150 cells transfected with antagomir-20b or its negative control (antagomir-NC) on the right flank (n = 5 mice/group). Tumor volume (V) was monitored by measuring the length (L) and width (W) of tumors with a caliper, and calculated with a formula V = π/6 (L × W)^3/2^. (C) Average weight of tumor tissues. After 40 days, the mice were sacrificed, and the tumor samples were collected and weighted. (D) qRT-PCR analyses of miR-20b expression in tumor tissues. (E) PTEN expression was detected by immunohistochemical staining. The data represent the mean ± SD. * *P* < 0.05, and ** *P* < 0.01, agomir-20b vs agomir-NC or antagomir-20b vs antagomir-NC.

## Discussion

It is well-known that microRNAs can regulate the expression of many genes involved in the initiation and maintenance of human diseases. In recent years, many microRNAs including miR-20b have been widely investigated as possible key regulators in the process of esophageal cancer development and treatment responses. MiR-20b belongs to the miR-106b-25 clusters, together with miR-17-92 and miR-106b-25 clusters, forms a large family called the miR-17 family [23]. The expression levels of miR-20b have been found to be upregulated in hepatocellular carcinoma [24], gastric cancer [14], and breast cancers [13]. In the present study, we firstly investigated the levels of miR-20b in the esophageal tumor tissues from clinical samples, we found that miR-20b expression was markedly elevated in the majority of esophageal tumor tissues compared with their neighboring normal tissues. although no statistical significant correlation was found between miR-20b expression and age, gender and tumor size, tumor differentiation degree, invasion depth, TNM stage and lymph node metastasis were found to significantly correlated with higher expression level of miR-20b, which suggests aberrant expression of miR-20b plays an important role in the development and progression of esophageal cancer. Further investigation revealed an inverse level of miR-20b expression and PTEN protein expression in the clinical samples. Additionally, we also studied the functional role of miR-20b and its possible mechanisms in regulating some biological properties of esophageal cancer cells. Our data showed that the differential expression of endogenous miR-20b was observed in various esophageal cancer cells, and its expression levels were relatively higher in lowly-differentiated cells, such as KYSE-150 and SKGT-5 cells compared with highly-differentiated cells, such as Eca-109, TE-1, and EC9706 cells. These findings suggest that miR-20b is associated with the differentiation degrees of esophageal cancer cells. A recent study indicated that miR-20 overexpression promoted the differentiation in embryo-derived mouse teratocarcinoma P19 cells by activating BMP signaling pathway [25]. However, another investigation demonstrated that overexpression of miR-20b repressed Th17 cell differentiation by targeting RAR-related orphan receptor γt (RORγt) and signal transducer and activator of transcription 3 (STAT3) [26]. Giraud-Triboult *et al*. found that the downregulation of miR-20b in mesenchymal stem cells (MSCs) leads to the overexpression of transcription regulator hypoxia-inducible factor 2α that participates in the determination of MSCs phenotype [27]. One of the reasons accounting for these discrepancies are possibly that there are different binding targets of miR-20b in various cells.

Based on expression pattern of miR-20b, we chose Eca-109 and KYSE-150 cells for the functional analysis of miR-20b through its overexpression and underexpression, respectively. Our results indicated that the upregulation of miR-20b in Eca-109 cells significantly promoted cell proliferation, migration, and invasiveness, and decreased the percentage of apoptotic cells in vitro. However, the forced overexpression of PTEN in these cells by transfection with PTEN expressing vector attenuated the abilities of cell migration and invasion, and augmented cellular apoptosis. On the other hand, downregulation of miR-20b in KYSE-150 cells inhibited cell viability, reduced cell migration and invasion abilities, and augmented apoptotic rate. But silenced PTEN expression in these cells by using PTEN siRNA increased the abilities of cell migration and invasion, and reduce apoptotic occurrence. These findings indicated that miR-20b-mediated effects on esophageal cells could be rescued by the cotransfection of PTEN expressing vector or PTEN siRNA. The results suggest that miR-20b-induced effects on esophageal cancer cells is closely associated with PTEN expression. Previous studies have demonstrated that miR-20b has an oncogenic role in breast cancer cells [28,21], gastric cancer [14], and colorectal cancer [29]. We further explored the biological significance of miR-20b in a xenograft model of nude mice. The results indicated that miR-20b expression upregulation promoted tumor growth, but its expression downregulation attenuated tumor growth in the mice. An inverse level of miR-20b and PTEN protein was observed in the tumor samples of mice.

PTEN is one of the most common tumor suppressors frequently mutated in human cancers, and it is a lipid phosphatase that cleaves the D3 phosphate of the second messenger phosphatidylinositol 3, 4, 5-trisphosphate and thus negatively regulates the phosphatidylinositol 3'-kinase (PI3K) pathway [30–32]. Previous studies have demonstrated that PTEN regulates not only cell cycle progress and apoptosis, but also cell migration, spreading, and focal adhesion formation [33]. Loss of PTEN was found to promote transforming growth factor beta-mediated cell motility and invasion [34]. Sawai *et al*. confirmed that loss of PTEN expression was involved in colorectal cancer aggressive capacity and liver metastasis [35]. Therefore, PTEN is an attractive target for anti-cancer therapy. PTEN expression can be regulated by miRNAs in various cancers, including hepatocellular carcinoma [36], glioma [37], ovarian cancer [38], and colorectal carcinoma [17]. A recent study showed that miR-20b could reduce PTEN protein expression by directly targeting the 3'-UTR of PTEN, and miR-20b was frequently overexpressed in breast cancer tissues and cell lines, and its expression upregulation significantly promoted the proliferation, colony formation and DNA synthesis in breast cancer cells [21]. In the present study, we found that PTEN is one of targets of miR-20b in esophageal cancer cells. The luciferase reporter assays confirmed that PTEN downregulation was mediated by the direct binding of miR-20b to the 3'-UTR of PTEN. This effect was abolished by the alteration of PTEN 3'-UTR region. Further investigation demonstrated that alteration of miR-20b expression only changed PTEN protein expression but not mRNA level. Therefore, we proposed that the main mechanism of miR-20b-induced PTEN downregulation was at posttranscriptional level, which is in agreement with previous reports [21].

Akt is a major downstream effector of PI3K pathway, and it has been shown to regulate cell proliferation and survival, and inhibits apoptosis through the regulation of downstream proteins [39]. Thus, PTEN expression downregulation can activate PI3K-Akt signaling pathway, which is associated with the development of cancers [40]. In the present study, upregulation of miR-20b reduced the level of PTEN protein in the Eca-109 cells, and simultaneously elevated p-Akt protein level, although it did not alter the level of Akt protein. By contrast, suppression of miR-20b expression increased PTEN protein level in the KYSE-150 cells, and synchronously reduced p-Akt protein expression. These results indicate miR-20b exerts its functional role possibly through regulation PTEN expression and PI3K/Akt signaling pathway.

In conclusion, our data indicate that miR-20b serves as an oncomir, and plays important roles in the regulation of some biological properties of esophageal carcinoma cells possibly by targeting tumor suppressor PTEN protein expression. Notably, our data showed that the upregulation of miR-20b promoted cell proliferation, migration, invasion, and tumor growth in vivo, and reduced apoptosis in the esophageal cancer cells. Conversely, miR-20b downregulation inhibited these processes in the esophageal cancer cells. Additionally, our data demonstrated that miR-20b negatively regulated PTEN expression only at the posttranscriptional level by directly binding the 3'-UTR of PTEN. Therefore, these findings suggest that miR-20b may be a novel diagnostic marker and potential therapeutic target for esophageal cancer treatment.
